RETRACTED

# Role of p38–MAPK pathway in the effects of high-magnitude compression on nucleus pulposus cell senescence in a disc perfusion culture

**DOI:** 10.1042/BSR20170718

**Published:** 2017-10-11

**Authors:** Lianglong Pang, Pei Li, Ruijie Zhang, Yuan Xu, Lei Song, Qiang Zhou

**Affiliations:** 1 Department of Spine Surgery, Liaocheng People's Hospital, Liaocheng, Shandong, 25200, China; 2 Department of Orthopedic Surgery, Southwest Hospital, Third Military Medical University, Chongqing 400038, China; 3 Department of Orthopedic Surgery, No.89 Hospital of PLA, Weifang, Shandong, 261026, China; 4 Department of Respiratory Medicine, The Third Xiangya Hospital, Central South University, Changsha, Hunan 410013, China; 5 Department of Orthopedic Surgery, Xinqiao Hospital, Third Military Medical University, Chongqing 400037, China

**Keywords:** intervertebral disc, nucleus pulposus, senescence, compression, p38-MAPK

## Abstract

Nucleus pulposus (NP) cell senescence is a typical pathological feature within the degenerative intervertebral disc. As a potential inducing and aggregating factor of disc degeneration, mechanical overloading affects disc biology in multiple ways. The present study was to investigate the NP cell senescence-associated phenotype under intermittent high compression in an *ex vivo* disc bioreactor culture, and the role of the p38–MAPK pathway in this regulatory process. Porcine discs were cultured in culture chambers of a self-developed mechanically active bioreactor and subjected to different magnitudes of dynamic compression (low-magnitude and high-magnitude: 0.1 and 1.3 MPa at a frequency of 1.0 Hz for 2 h per day respectively) for 7 days. Non-compressed discs were used as controls. The inhibitor SB203580 was used to study the role of the p38–MAPK pathway in this process. Results showed that intermittent high-magnitude compression clearly induced senescence-associated changes in NP cells, such as increasing β-galactosidase-positive NP cells, decreasing PCNA-positive NP cells, promoting the formation of senescence-associated heterochromatic foci (SAHF), up-regulating the expression of senescence markers (p16 and p53), and attenuating matrix production. However, inhibition of the p38–MAPK pathway partly attenuated the effects of intermittent high-magnitude (1.3 MPa) compression on those described NP cell senescence-associated parameters. In conclusion, intermittent high-magnitude compression can induce NP cell senescence-associated changes in an *ex vivo* disc bioreactor culture, and the p38–MAPK pathway is involved in this process.

## Introduction

Intervertebral disc degeneration is regarded as a major cause of lower back pain [1]. This physical disability products substantial economic burdens on social health care systems and great inconvenience to the daily activity of patients [2]. Despite the rapid progression in tissue engineering-based regenerative medicine and function reestablishment-based surgical therapy, the biological regeneration of degenerative discs remains a future goal.

RETRACTED

During disc degeneration, corresponding pathological changes first occur in the nucleus pulposus (NP) region, such as decreased matrix synthesis and increased cell apoptosis [3,4]. In the last decade, cellular senescence was systematically studied in human discs and reported to aggravate in degenerated discs [5–7]. Although senescent cells can remain viable for a long time, their morphology, and biological function largely differ from non-senescent cells. This transition into the senescent phenotype directly causes cell growth arrest and the imbalance between matrix catabolism and anabolism [8]. Based on these findings, it is reasonable to deduce that cell senescence may be involved in the disc degeneration process.

Intervertebral disc (IVD) is located between two adjacent vertebral bones and functions in load bearing, and absorbtion [9]. During daily activities, the IVD undergoes various magnitudes of mechanical load, which in turn affect disc cell viability and biological function [10–12]. It is well established that physiological mechanical loads are beneficial for disc biology, whereas non-physiological loads can initiate and accelerate disc degeneration [11–13]. Previously, a foreleg amputation-induced rat disc degeneration model showed increased senescent cells within the degenerative disc [14–16]. These studies indirectly indicated that excessive and continuous mechanical compression caused by prolonged upright postures may aggravate cellular senescence within the disc.

The intact disc organ culture system is an appropriate and common model to study NP biology because of its precise controllability over external stimuli and its retention of native structural integrity [17,18]. Additionally, the development of a bioreactor platform allows for disc organ culture study under near-physiological conditions [19]. Previously, we successfully established a porcine disc bioreactor culture system in which disc NP cell viability could be maintained for a long time [20]. Therefore, we mainly investigated the effects of high compressive strength on senescence-associated changes of NP cells using this porcine disc bioreactor culture system. Additionally, the role of the p38–MAPK signaling pathway in this process was studied using the specific inhibitor SB203580. The NP cell senescence phenotype was evaluated by SA-β-galactosidase staining, senescence-associated heterochromatic foci (SAHF), cell proliferation potency, and matrix protein metabolism.

RETRACTED

## Materials and methods

### Ethical statement

All animal experiments complied with relevant guidelines and regulations of the Ethics Committee at Southwest Hospital affiliated to the Third Military Medical University [SYXK (YU) 2012-0012].

### Bioreactor design

As illustrated in Figure 1, the perfusion bioreactor consists of a medium reservoir, peristaltic pump, substance exchanger, pH sensor, PO_2_ sensor, PCO_2_ sensor, tissue culture chamber, loading application device, and other ancillary equipment. Mechanical loading is axially applied with an integrated servomotor mated with the culture chamber and simultaneously adjusted by a central controller. The number of culture chambers can be adjusted according to the sample size and group number. The medium perfusion system includes two circulating loops: an incubation loop and a medium supplement loop. Fresh medium in the medium supplement loop can be recycled into the medium reservoir after flowing through the substance exchanger. Additional details about this bioreactor system have been reported previously [21].

**Figure 1:** Introduction of the perfusion bioreactor system. (**A**) Photograph of this substance exchanger-based perfusion bioreactor. (**B**) The scheme of this novel bioreactor system (1: medium reservoir; 2: substance exchanger; 3: peristaltic pump; 4: tissue culture chamber; 5: pH, PO_2_ and PCO_2_ sensor).

### Disc harvest and bioreactor culture

Twelve healthy pigs (3–4 months old) used in the present study received standard housing and husbandry the Animal Center of Third Military Medical University. Briefly, after the animals were anesthetized with pentobarbital sodium, the spinal column was isolated under sterile conditions. Then, the ligaments and connective tissues were removed, and discs (T11/12-L4/5) with cartilage endplate (CEP) were separated and rinsed with phosphate buffer saline (PBS) as described previously [22]. After the disc area (Area ≈ π(*W*_ap_*W*_lat_)/4, where *W*_ap_ and *W*_lat_ are the anterior-posterior and lateral widths respectively) was measured to calculate the compressive magnitude [23], the discs were cultured for 7 days using our self-developed bioreactor and randomly assigned to different intermittent compression groups (0.1 and 1.3 MP at a frequency of 1.0 Hz for 2 h once per day). When the application of compression was finished, all discs in the compression groups (0.1 and 1.3 MPa) were perfusion-cultured in the same medium during the remaining 22 h of the day. Discs without intermittent compression were used as controls and cultured under the same conditions. To investigate the role of the p38–MAPK pathway in the effects of intermittent high-magnitude (1.3 MPa) compression on NP cell senescence, the discs from the 1.3 MPa group were pretreated with the inhibitor SB203580 (10 μM in  dimethyl sulfoxide (<0.1%), which was determined from a previous study and our own experience [24]) that was added along with the culture medium. Fresh DMEM/F12 culture medium (HyClone, U.S.A.) supplemented with 10% (v/v) FBS (Gibco, U.S.A.) and 1% (v/v) penicillin–streptomycin (Gibco, U.S.A.) was circulated at a rate of 5 ml/min. To decrease the interference caused by the difference between different disc levels, the three discs from the same levels (e.g. T11/T12, T12/L1, and L1/L2) of different animals were used for the same assay in each group, which was also described previously [25].

RETRACTED

### SA-β-galactosidase staining assay

After culture, central NP tissues were immediately separated from discs (T11/T12, T12/L1, and L1/L2) under a dissecting microscope. Then, NP cells were isolated by enzymatic digestion with 0.25% trypsin for 5–10 and 0.25% Type I collagenase (Sigma) for 30 min at 37°C. Thereafter, cell pellets were resuspended in a monolayer culture and cultured for an additional 4 h to allow cell attachment under standard conditions (37°C, 21% O_2_ and 5% CO_2_). Then, SA-β-galactosidase staining was performed using a Senescence β-Galactosidase Staining Kit (Beyotime, China) according to the manufacturer’s instructions. SA-β-galactosidase-positive NP cells were observed under a light microscope (Olympus BX51) and analyzed using Image-Pro Plus software (Version 5.1, Media Cybernetics, Inc.). SA-β-galactosidase activity was expressed as the percentage of NP cells staining positive among all NP cells.

### Alcian Blue staining assay

After discs (L2/L3, L3/L4, and L4/L5) were sequentially fixed with 4% paraformaldehyde, decalcified with 10% ethylenediaminetetraacetic acid (EDTA) and embedded in paraffin, 5-μm thick cross-sections were prepared. To generally observe proteoglycan (PG) distribution in the NP tissue, Alcian Blue staning was performed. All sections were observed under a light microscope (Olympus BX51) using the same photo parameters. The staining intensity was expressed as IOD and was analyzed using Image-Pro Plus software (Version 5.1, Media Cybernetics, Inc.) with the same linear calibration.

### SAHF observation

Disc sections (L2/L3, L3/L4, and L4/L5) prepared in the Alcian Blue staining assay were used to analyze SAHF development. Briefly, the 5-μm thick sections were deparaffinized and stained with DAPI solution (Beyotime, China) for 10 min at room temperature. Then, sections were viewed under a laser scanning confocal microscope (Zeiss, LSM780, Germany) and analyzed using the Image-Pro Plus software (Version 5.1, Media Cybernetics, Inc.). The percentage of SAHF-positive NP cells to the total NP cells was used to reflect NP cell senescence.

RETRACTED

### Real-time PCR analysis

Real-time PCR was performed to analyze mRNA expression of matrix molecules (aggrecan and collagen II), matrix remodeling enzymes (TIMP-1, TIMP-3, ADAMTS-4, and MMP-3) and senescence-related markers (p16 and p53). Briefly, after total RNA was extracted with TRIzol reagent (Invitrogen, U.S.A.) from the isolated central NP tissue (L2/L3, L3/L4, and L4/L5), 1 μg of RNA in each group was used for a cDNA synthesis assay using a reverse transcription kit (Roche, Switzerland). Then, the primers (Table 1), cDNA samples, and SYBR Green qPCR Mix (DONGSHENG BIOTECH, China) were mixed together and subjected to a real-time PCR reaction. Fresh disc NP samples were used as controls, and GAPDH was used as the reference gene. The relative expression of target genes was expressed as 2^−ΔΔ*C*^_T_.

**Table 1:** Primers of target genes

Gene	Accession number	Forward (5′–3′)	Reverse (5′–3′)
GAPDH	NM_001206359.1	ACCTCCACTACATGGTCTACA	ATGACAAGCTTCCCGTTCTC
Aggrecan	NM_001164652.1	CGTGGTCCAGCACTTCTAAA	AGTCCACTGAGATCCTCTACTC
Collagen II	XM_001925959.4	CCGGGTGAACGTGGAGAGACTG	CGCCCCCACAGTGCCCTC
ADAMTs-4	XM_003481414.2	TTCAACGCCACGTTCTACTC	GCCGGGATGATGAGGTTATTT
MMP-3	NM_001166308.1	GCCCGTTGAGCCCACAGAATCTAC	GGAAGAGGTGGCCAAAATGAAGAG
TIMP-1	NM_213857.1	CCTGACATCCGGTTCATCTA	CAGTTGTCCAGCTATGAGAAAC
TIMP-3	XM_003126073.4	GGATTGTGTAACTTTGTGGAGAG	GGCAGGTAGTAGCAGGATTTA
P16	XM_013993499.1	TGCAGTTGCCTACCTCTGAA	CGAATCCGCACAGTAATCAA
P53	NM_213824.3	CCTTAAGATCCGTGGGCGT	GCTAGCAGTTTGGGCTTTCC
P21	XM_013977858.2	CCTCTAAGGTTGGGCAGGGT	TTTCACTGGACAGAGGGGCT

### Western blotting assay

The expression of p38 MAPK, phosphor-p38 MAPK, p16, and p53 protein was evaluated by western blot. Briefly, after total protein was extracted with RIPA lysis solution (Beyotime, China) from the isolated central NP tissue (T11/T12, T12/L1, and L1/L2), protein samples were subjected to the SDS/PAGE system and transferred onto PVDF membranes, followed by incubation with primary antibodies (p38–MAPK: Cell Signaling Technology, #14451; phospho–p38–MAPK: Cell Signaling Technology, #4092; p53: Biosource, #MBS8242548; p16: Santa Cruz, sc-28260; p21: Santa Cruz, sc-397; β-actin: Proteitech, 60008-1-Ig) at 4°C overnight and incubation with the corresponding HRP-conjugated secondary antibodies (goat anti-mouse IgG and goat anti-rabbit IgG, ZSGB-BIO, China, diluted 1:2000) at 37°C for 2 h. Then, protein bands on the PVDF membrane were detected using a SuperSignal West Pico Trial Kit (Thermo) and analyzed using ImageJ software (National Institutes of Health, U.S.A.) to obtain the gray value for each band. The expression of target protein (p16 and p53) was normalized to that of β-actin. The expression of p38–MAPK was normalized to that of p–p38–MAPK to reflect p38–MAPK pathway activity.

RETRACTED

### Immunohistochemical staining

To analyze matrix protein deposition within the NP region and NP cell proliferation potency, immunohistochemical staining of macromolecules (aggrecan and collagen II) and proliferating cell nuclear antigen (PCNA) respectively, were performed on disc sections (L2/L3, L3/L4, and L4/L5) as described previously [11]. The primary antibodies used in the present study were rabbit anti-collagen II polyclonal antibody (Abcam, diluted 1:200), mouse anti-aggrecan monoclonal antibody (Norvus, NB120-11570, diluted 1:400), and mouse anti-PCNA monoclonal antibody (Proteintech, 60097-1-Ig, diluted 1:200). Once the disc sections were reacted with HRP-conjugated secondary antibodies (goat anti-mouse IgG and goat anti-rabbit IgG, ZSGB-BIO, China, diluted 1:200), diaminobenzidine (DAB) was used for color development. Finally, all sections were observed under a light microscope (Olympus BX51) using the same photo parameters. The staining intensity was expressed as integral optical density (IOD), which was analyzed using Image-Pro Plus software (Version 5.1, Media Cybernetics, Inc.) with the same linear calibration.

### Biochemical content measurement

After compression culture, NP tissues (L2/L3, L3/L4, and L4/L5) were isolated and prepared for the quantification of glycosaminoglycan (GAG) and hydroxyproline (HYP) content. Briefly, NP tissues used for GAG content measurement were lyophilized for 24 h and immediately weighed to obtain the dry weight, followed by the papain digestion procedure at 60°C for 24 h. Then, GAG content (μg/mg dry weight) was determined according to the absorbance value at a wavelength of 525 nm and the standard curve created by gradient concentrations of shark cartilage chondroitin sulfate using the dimethyl methylene blue (DMMB) method [26]. NP tissues for HYP content measurement were immediately weighted to determine their wet weight after isolation. Then, after NP samples were incubated with hydrolysate, HYP content was analyzed using an HYP quantification kit (Nanjing Jiancheng, China) according to the manufacturer’s instructions.

### Statistics

All numerical data in the present study were presented as the mean ± S.D. and analyzed for statistical difference using the SPSS 13.0 software. Each experiment in this work was performed in triplicate. In the present study, when a homogeneity test for variance was completed, one-way analysis of variance (ANOVA) was performed, and then a post hoc LSD test was performed. A statistical difference was indicated when the *P*-value <0.05.

RETRACTED

## Results

### Analysis of p38–MAPK pathway activity

To investigate whether the p38–MAPK pathway in NP cells was activated under intermittent compression, the relative expression of phospho–p38–MAPK to total p38–MAPK was analyzed. Results showed that p38–MAPK pathway activity in the 1.3 MPa group was significantly increased compared with that in the 0.1 MPa group and the control group (Figure 2A). To verify whether the p38–MAPK pathway participated in the described effects of intermittent high-magnitude compression on NP cell senescence, the inhibitor SB203580 effectively inhibited activation of the p38–MAPK pathway both in the control group and the 1.3 MPa+SB group (Figure 2B).

**Figure 2:** PI3K/Akt pathway activity analysis. Analysis of p38–MAPK pathway activity in NP cells of porcine discs subjected to different magnitudes of compression. (**A**) High-magnitude (1.3 MPa) compression significantly increased p38 pathway activity compared with the low-magnitude (0.1 MPa) compression. (**B**) The inhibitor SB203580 clearly inhibited activation of p38–MAPK pathway in NP cells both in the control group and the high-magnitude (1.3 MPa) compression group. The data are expressed as the means ± S.D., *n*=3. #: indicates a significant difference compared with the control group. *: indicates a significant difference between two groups (*P*<0.05).

### SA-β-galactosidase staining and formation of SAHF

As shown in Figure 3(A), senescent NP cells were found in the NP region in each group (shown by arrows). Though a significant difference between the 0.1 MPa group and control group was not found, the 1.3 MPa group showed a higher percentage of SA-β-galactosidase-positive NP cells than the control group and 0.1 MPa group. Inhibition of p38–MAPK pathway decreased the number of SA-β-galactosidase-positive NP cells in the 1.3 MPa group. However, the number of SA-β-galactosidase-positive NP cells in the 1.3 MPa+SB group was higher than in the control or 0.1 MPa group. As shown in Figure 3(B), SAHF measurements revealed a similar trend before and after inhibition of the p38–MAPK pathway among these groups.

**Figure 3:** Senescence-associated staining observation. SA-β-galactosidase staining (**A**) and SAHF formation (**B**) in NP cells of porcine discs subjected to different compression magnitudes. The data are expressed as the means ± S.D., *n*=3. # and &: indicate a significant difference compared with the control and 0.1 MPa groups respectively. *: indicates a significant difference between two groups (*P*<0.05).

RETRACTED

### Expression of senescence markers

As both the p53–p21–pRb and p16–pRb pathways are well known to be related to cellular senescence [5], we evaluated the effects of mechanical compression on p16, p21, and p53 expression both at the gene and protein levels. As shown in Figure 4, though expression of p16, p21, and p53 were similar between the control group and 0.1 MPa group, the 1.3 MPa group exhibited a significantly up-regulated expression of p16, p21, and p53 compared with both the control group and the 0.1 MPa group. Similarly, the inhibitor SB203580 decreased the expression of p16, p21, and p53 under 1.3 MPa dynamic compression. However, expression of p16 and p53 in the 1.3 MPa+SB group were higher than in the control group.

**Figure 4:** Analysis of senescence markers expression. Expression of senescence markers (p16, p21, and p53) in NP cells of porcine discs subjected to different compression magnitudes. (**A**) Real-time PCR analysis of p16, p21, and p53 gene expression. (**B**) Western blot analysis of p16, p21, and p53 protein expression. The data are expressed as the means±S.D., *n*=3. # and &: indicate a significant difference compared with the control and 0.1 MPa groups respectively. *: indicates a significant difference between two groups (*P*<0.05).

### Gene expression of matrix metabolism-related molecules

In the present study, we analyzed gene expression of matrix macromolecule genes (aggrecan and collagen II) and matrix remodeling genes (ADAMTS-4, MMP-3, TIMP-1, and TIMP-3). Results showed that intermittent high compression (1.3 MPa) significantly down-regulated the expression of aggrecan, collagen II and TIMP-3 mRNA, but up-regulated the expression of matrix degradation-related enzymes (ADAMTS-4 and MMP-3) compared with the control group and intermittent low compression (0.1 MPa). In contrast, low compression (0.1 MPa) significantly up-regulated the expression of aggrecan, collagen II, and TIMP-3 and down-regulated MMP-3 mRNA compared with the control group. TIMP-1 mRNA expression showed no difference among the control, 0.1 and 1.3 MPa groups. However, when the inhibitor SB203580 was applied to the 1.3 MPa group, the expression of aggrecan and collagen II genes was partly up-regulated, whereas the expression of ADAMTS-4 and MMP-3 genes was clearly down-regulated in the high-magnitude (1.3 MPa) compression group (Figure 5).

**Figure 5:** Expression of matrix remodeling-associated molecules. Real-time PCR analysis of matrix molecule (aggrecan and collagen II) expression and matrix remodeling enzyme (ADAMTS-4, MMP-3, TIMP-1, and TIMP-3) expression in NP cells of porcine discs subjected to different compression magnitudes. The data are expressed as the means ± S.D., *n*=3. # and &: indicate a significant difference compared with the control and 0.1 MPa groups respectively. *: indicates a significant difference between two groups (*P*<0.05).

RETRACTED

### Matrix production

The extracellular matrix of disc NP tissue is rich in PGs, which can be stained by Alcian Blue. As shown in Figure 6(A), Alcian Blue staining intensity in the 0.1 MPa group was higher than in the control group. However, the intermittent high-magnitude (1.3 MPa) compression group showed a significant decrease in staining intensity compared with the control and 0.1 MPa groups, indicating that the PG content was dramatically reduced under high-magnitude compression. However, Alcian Blue staining intensity in the 1.3 MPa group was significantly increased by the inhibitor SB203580.

**Figure 6:** Matrix production analysis. Matrix production of NP cells of porcine discs subjected to different compression magnitudes. (**A**) Alcian blue staining assay. (**B**) Immunostaining of aggrecan and collagen II; magnification: 200×, scale = 100 μm. (C) Measurement of GAG and HYP levels. The data are expressed as the means ± S.D., *n*=3. # and &: indicate a significant difference compared with the control and 0.1 MPa groups respectively. *: indicates a significant difference between two groups (*P*<0.05).

To evaluate matrix protein expression in the NP region, we observed immunostaining of aggrecan and collagen II in the present study. Results showed that 1.3 MPa compression decreased the staining intensity of both aggrecan and collagen II compared with the 0.1 MPa compression and the control group, whereas the 0.1 MPa compressive strength increased aggrecan and collagen II staining intensity compared with the control group. However, when p38–MAPK activation was inhibited by inhibitor SB203580, the staining intensity of these matrix proteins (aggrecan and collagen II) in the 1.3 MPa group was partly increased (Figure 6B).

We also measured GAG and HYP levels to evaluate NP matrix metabolism. Results showed that both GAG and HYP levels were decreased in the 1.3 MPa group compared with the 0.1 MPa group and the control group, whereas GAG and HYP levels in the 0.1 MPa group were increased compared with the control group. Additionally, the inhibitor SB203580 partly increased GAG and HYP levels within the disc NP region under 1.3 MPa compression (Figure 6C).

### Immunohistochemistry for PCNA

NP cell proliferation was evaluated by PCNA immunostaining. In the present study, although the percentage of PCNA immuno-positive NP cells was similar between the control and 0.1 MPa groups, it was clearly decreased in the 1.3 MPa compression group. However, the p38–MAPK inhibitor SB203580 attenuated intermittent high-magnitude (1.3 MPa) compression-induced effects on PCNA immunostaining. Additionally, the percentage of PCNA immuno-positive NP cells in the 1.3 MPa+SB group was lower than in the control or 0.1 MPa group (Figure 7).

RETRACTED

**Figure 7:** Analysis of PCNA expression. PCNA immunohistochemistry in NP tissue of porcine discs subjected to different compression magnitudes; magnification: 200×, scale = 100 μm. The data are expressed as the means ± S.D., *n*=3. # and &: indicate a significant difference compared with the control and 0.1 MPa groups respectively. *: indicates a significant difference between two groups (*P*<0.05).

## Discussion

Cellular senescence is an important mechanism that regulates age-related dysfunctions and chronic disease [27]. Recently, senescent cells have also been identified as a classical pathology in degenerative human and animal discs [5,6]. Importantly, several studies have demonstrated that cellular senescence plays an important role in the disc degeneration process [7,28]. Mechanical compression significantly affects disc NP cell biology *in vivo* and *in vitro* [13,24]. In the present study, we studied the effect of mechanical compression on NP cell senescence in an *ex vivo* disc bioreactor culture. Our results demonstrated that intermittent high compression could significantly induce senescence-associated changes in disc NP cells compared with intermittent low compression. However, the inhibition of p38–MAPK partly attenuated the effects of intermittent high compression on NP cell senescence. The present study provides a mechanism by which excessive mechanical load initiates and/or aggravates the disc degeneration process.

β-Galactosidase staining and SAHF observation are useful and common methods for identifying cellular senescence [29,30]. Furthermore, senescent cells are often arrested in the G1–S cell cycle transition, which leads to limited cell proliferation potency [31]. PCNA is a useful marker to evaluate cell proliferation [32]. In the present study, we found that intermittent high-magnitude (1.3 MPa) compression increased the number of β-galactosidase-positive and SAHF-positive NP cells, but decreased the number of PCNA immuno-positive NP cells compared with intermittent low-magnitude (0.1 MPa) compression and the control group. All these results indicate that intermittent high-magnitude compression promotes NP cell senescence compared with intermittent low-magnitude compression. In line with this to some extent, a study on the disc degeneration model induced by foreleg amputation demonstrated that disc cell senescence could be accelerated by mechanical overloading, which was caused by forelimb-amputation-induced prolongation of upright postures.

RETRACTED

Two mechanisms are responsible for the induction of cellular senescence: the replicative senescence (RS) mediated by the p53–p21–pRB pathway and stress-induced premature senescence (SIPS) mediated by the p16–pRB pathway [5]. Activation of the p53–p21–pRB or p16–pRB pathway depends on the stimulus type and the resulting changes in the microenvironment surrounding disc cells [27]. In the present study, the expression of p16, p21, and p53 in the intermittent high-magnitude (1.3 MPa) compression group was higher than in the intermittent low-magnitude (0.1 MPa) compression group and control group, indicating that intermittent high-magnitude (1.3 MPa) compression may accelerate premature senescence of NP cells through the RS and SIPS approaches. In line with this, a previous study demonstrated that p16 and p53, though uncommon, are co-expressed in the disc tissue of some patients [33], further supporting the hypothesis that there are situations in which the RS and SIPS pathways are activated simultaneously.

Although senescent cells become unresponsive to mitogenic stimuli, they can remain alive and exhibit catabolism-like matrix metabolism [27]. A previous study using the bovine disc organ culture system demonstrated that senescent disc NP cells induced by the inflammatory cytokine TNF-α have a reduced anabolic metabolism characterized by increased aggrecan degradation products and down-regulated matrix macromolecule (aggrecan, collagen I, and collagen II) expression [34]. In our previous work, we also found that senescent cells exhibited an attenuated matrix anabolic metabolism [35,36]. Here, matrix homeostatic phenotype was used as a indirect parameter for evaluating NP cell senescence. We found that attenuated NP matrix biosynthesis is accompanied by promoted NP cell senescen in the intermittent high-magnitude (1.3 MPa) group. On one hand, the attenuated matrix biosynthesis may be resulted from the high-magnitude compression, which has been confirmed by previous studies [37,38]. On another hand, it may also be the secondary consequence of high-magnitude compression-induced NP cell senescence.

The p38–MAPK pathway converts extracellular stimuli into cellular biological responses to regulate cellular bioactivities including apoptosis, proliferation, and senescence [39]. Previous studies have reported that mechanical stimuli can activate the p38–MAPK signaling pathway in chondrocytes [40–42]. In line with this, we found that the p38–MAPK pathway in disc NP cells was activated under mechanical compression. Moreover, the activity of p38 activity in the 1.3 MPa group was clearly higher than in the 0.1 MPa and control groups, indicating that the p38–MAPK pathway may be involved in certain effects of high-magnitude (1.3 MPa) compression on disc NP cells. Our subsequent analysis showed that the inhibition of p38–MAPK in the 1.3 MPa group clearly attenuated the effects of intermittent high-magnitude (1.3 MPa) compression on NP cell senescence-associated parameters (1.3 MPa group versus 1.3 MPa+SB group), such as SA-β-galactosidase staining, the formation of SAHF, senescence marker (p16 and p53) expression, PCNA immunostaining and the matrix homeostatic phenotype. This suggests that the p38–MAPK pathway is partly involved in the promotive effects of intermittent high-magnitude compression on disc NP cell senescence.

RETRACTED

The present study also has several limitations. First, although porcine discs have been used to study disc biology in many studies [43–45], results in the present study may have limited stringency in reflecting the mechanobiology of the adult disc because the immature porcine disc contains a high content of notochordal cells that were disappeared in adult human discs [46,47]. Second, although we verified the role of the p38–MAPK pathway in the high-magnitude compression-induced disc NP cell senescence using the inhibitor SB203580, a more specific inhibitor UR-13756 used in a previous study [48] or a genetic animal model with kinase-knockdown may further strengthen our results.

Based on the results from the present study, we conclude that intermittent high-magnitude compression can induce disc NP cell senescence in an *ex vivo* disc organ culture, and that the p38–MAPK pathway may participate in this regulatory process. The present study demonstrates that external excessive mechanical compression may gradually induce disc NP cell senescence and result in destructive effects on NP matrix remodeling and thus contribute to disc degeneration.

## Abbreviations

ADAMTS-4: a disintegrin and metallopeptidase with thrombospondin motifs 4
DMEM/F12: dulbecco's modified eagle media: nutrient mixture F-12
GAG: glycosaminoglycan
HRP: horseradish peroxidase
HYP: hydroxyproline
IOD: integral optical density
IVD: intervertebral disc
LSD: least significant difference
MMP-3: matrix metalloproteinase 3
NP: nucleus pulposus
PCNA: proliferating cell nuclear antigen
RIPA: radio-immunoprecipitation assay
RS: replicative senescence
SAHF: senescence-associated heterochromatic foci
SIPS: stress-induced premature senescence
TIMP-1: tissue inhibitor of metalloproteinase-1
TIMP-3: tissue inhibitor of metalloproteinase-3
TNF-a: tumor necrosis factor-a
qPCR: quantitative polymerase chain reaction
